# Thymol Disrupts Cell Homeostasis and Inhibits the Growth of *Staphylococcus aureus*

**DOI:** 10.1155/2022/8743096

**Published:** 2022-08-13

**Authors:** Qingxiang Li, Ke Xing Huang, Sheng Pan, Chun Su, Juan Bi, Xuan Lu

**Affiliations:** ^1^Department of Newborn, Affiliated Hospital of Zunyi Medical University, Zunyi, Guizhou 563000, China; ^2^Department of General Medicine, Shenzhen Longhua District Central Hospital, Shenzhen, Guangdong 518000, China; ^3^Center for Excellence in Molecular Cell Science, Chinese Academy of Sciences, University of Chinese Academy of Sciences, Shanghai 210000, China; ^4^Department of Pharmacy, Shanghai Changhai Hospital, Naval Medical University, Shanghai, China; ^5^School of Life SNciences, Hefei Nomal University, Hefei, Anhui 230031, China

## Abstract

*Staphylococcus aureus* (*S. aureus*) is a typical kind of symbiotic bacteria, which can cause human pneumonia, food poisoning, and other health problems. Nowadays, the corresponding prevention and treatment have been a hot issue of general concern in related research areas. However, the mechanism of action against *S. aureus* is not well understood. In order to tackle such problem, we used broth microdilution to discuss the antibacterial effect of 5-methyl-2-isopropylphenol and determine inhibitory concentration. In addition, membrane potential and lipid peroxidation levels were also measured under experimental conditions. The experimental results suggested that 300 *μ*g/mL thymol might cause cell membrane damage and decrease of NADPH concentration and increase of NADP^+^ and lipid peroxidation level. In such condition, thymol has the potential to result in membrane rupture and disruption of cellular homeostasis. Furthermore, we also found that NOX_2_ is involved in maintaining the balance of NADPH/NADP^+^ in cells. Finally, our work confirms that NOX_2_ is a potential downstream target for thymol in the cell. Such target can provide specific guidance and recommendations for its application in antifungal activity. Meanwhile, our study also provides a new inspiration for the molecular mechanism of thymol's bacteriostatic action.

## 1. Introduction

*Staphylococcus aureus* (*S. aureus*) is both a commensal and opportunistic bacterium, causing a variety of infections in humans, such as bacteremia, pneumonia, skin and soft tissue infections, and food poisoning [1–4]. It was recently suggested to be the major cause of late-onset sepsis in very-low birth weight infants admitted to neonatal intensive care units in the USA and UK [5–7]. Data from 2005 to 2018 suggested that up to 4.4% of very-low birth weight infants in China developed *S. aureus* bacteremia or meningitis and osteomyelitis, with an overall mortality of 19% to 30.5% [8–12]. Moreover, a recent meta-analysis showed that the risk of *S. aureus* colonization and infection in infants was 24.2 times higher than that in adults, indicating that infants were at high risk for *S. aureus* colonization [10, 13]. At the same time, a number of factors, including the mechanisms by which traditional antibiotics work, the misuse of antibiotics, and the lack of new targeted antibiotics, have led to an alarming rate of drug resistance and tolerance [14–16]. Therefore, the development of new prevention and treatment measures, including the identification of new targets for small molecule inhibitors, enzymes, and immunological drugs, to meet the growing challenge of *S. aureus* is our most urgent task at present.

5-Methyl-2-isopropylphenol (thymol) is a monoterpene phenol, which is mainly isolated from plants belonging to the Lamiaceae family including Thymus, Ocimum, Origanum, and Monardagenera [17–21]. thymol has been shown to possess antiseptic, antibacterial, antifungal, anthelmintic, antiviral, antioxidant, expectorant, antispasmodic, carminative, diaphoretic, sedative, antirheumatic, and even anticancer, antihyperlipidemic, and antihyperglycemic action [16, 22–26]. Coppo and Marchese [27] revealed that the antibacterial activity of essential oil containing thymol (32.55%) showed antibacterial activity against most Gram-positive and Gram-negative bacteria [27–29]. Reports from Olasupo summarized that the minimum inhibitory concentrations (MIC) of thymol were 1.0 *μ*mol/L for *S. typhimurium* (0.15 mg/mL), 1.2 *μ*mol/L for *Escherichia* (0.18 mg/mL), 2.0 *μ*mol/L for *S. aureus* (0.31 mg/mL), and 33 *μ*mol/L for *E. coli* (5.00 mg/mL), respectively [30–32]. The most commonly accepted explanation for the antimicrobial mechanism of thymol is that the changes in membrane tension caused by thymol destabilize membrane structure. The antibacterial mechanism of thymol showed that its ability to bind to the lipid layer of cell membrane increased its surface curvature. The hydrophilic part of the molecule interacts with the polar part of the membrane, while the hydrophobic benzene ring and lipid side chains sink into the inner layer of the biofilm. This has led to a dramatic change in membrane structure through the instability of the lipid layer, decreased elasticity, and increased fluidity [25, 33–35]. Several studies have currently shown that thymol can lead to the breakdown of adenosine triphosphate (ATP) synthesis, which disrupts the bioenergy balance and damages mitochondrial energy production. It may also cause metabolic disorders of Na^+^ and Ca^2+^ in cells to produce excessive oxygen free radicals, leading to cell death [36–38]. Therefore, application of thymol is considered as an efficient treatment for food preservation and control of microbial growth and infection [16, 39, 40]. Lin et al. [12] suggest that thymol/cyclodextrin-inclusion (CD-IC) can be used in the food industry as a food packaging and antibacterial agent [22]; Serna-Escolano et al. [41] found that 2-hydroxylpropyl-betacyclodextrin-thymol encapsulated by MW could be a promising alternative to synthetic fungicides for controlling *G. citri-aurantii*, the causal agent of citrus sour rot [41].

In this study, the antimicrobial effects of thymol against *S. aureus* were explored to elucidate its potential mechanism. Thymol related biofilm dysfunctions were studied by using Scanning Electron Microscopy (SEM) to detect the changes in cell membrane potential, intracellular NADPH/NADP^+^, ATP concentrations, and membrane integrity. Moreover, the MDA concentration is also discovered as an indicator to track the oxidation level of cell membranes. This study will encourage people to use thymol as a natural antibacterial agent in their daily life.

## 2. Materials and Methods

### 2.1. Reagents

The stock solution of thymol (T118449, ≥99.9% (GC)) was purchased from the Aladdin Biochemical Technology Co., Ltd (Shanghai, China). Unless otherwise noted, thymol solutions in different concentrations used under all conditions were prepared by mixing medium (Cation-Adjusted Mueller-Hinton II Broth (CA-MHII) or Tryptone Soya Broth (TSB)), PBS, and 2.5% (v/v) ethanol. Propidium iodide (PI) staining solution (1 mg/mL; Yeasen, Shanghai, China) was used to measure membrane destruction. These solutions were sterilized using a 0.22 *μ*m filter and were stored at −20°C until analysis. Lipid Peroxidation (MDA) Assay Kit (ab118970) and Cellular Membrane Potential Assay Kit (ab176765) were purchased from Abcam Co., Ltd. All other chemicals used to configure various buffers were maintained in the analytical grade and purchased from the Aladdin Biochemical Technology Co., Ltd (Shanghai, China).

### 2.2. Bacterial Strain and Culture Conditions

*S. aureus* ATCC25923 and ATCC43300 were purchased from American Type Culture Collection (ATCC; Manassas, VA, USA). *S. aureus* RN4220 was purchased from Huayueyang biotech co. ltd (Beijing, China). To activate the strain, all purchased strains were activated for three generations before use to maintain good physiological status. During the activation process, all strains were inoculated into fresh TSB and replaced medium every 12 hours. After 36 h of incubation at 37°C, the bacteria grow to the logarithmic growth phase or kept stable at the stable phase. The strains used in the experiment were activated strains.

### 2.3. Inhibitory Concentration Determination

The inhibitory concentration of thymol against *S. aureus* was determined using broth microdilution method as described elsewhere [42]. Activated *S. aureus* ATCC25923 and ATCC43300 cells were obtained until OD_600_ = 0.5 (approximately 10^8^ CFU/mL) by using the method described in Section 2.2. The thymol solution was prepared at a concentration of 2.4 mg/mL and then diluted into ideal concentrations in CA-MHII medium at 0, 50, 100, 150, 200, 300, 400, 600, 800, and 1200 *μ*g/mL. The electron carrier solution was diluted 8-fold with sterile water, and the WST solution and the diluted electron carrier solution were prepared in a ratio of 9 : 1. The cell suspension was diluted with sterile water to adjust the cell concentration to about 10^7^ CFU/mL. 10 *μ*l cell suspension and 180 *μ*l thymol solutions at different concentrations were added into each well to maintain a final cell density of 10^4^ CFU/ml. After incubation for 6 h, 10 *μ*L working solution was added to each well and incubated at 37°C for 2 h. For each concentration, microbial growth was determined by microplate reader at 600 nm.

### 2.4. Growth Curves

The optical density at 600 nm was measured every 1.0 hour using a full-wavelength scanning multifunction reader (Thermo Fisher, Finland) to monitor cell growth. Specifically, *S. aureus* ATCC25923 was grown to an OD600 value of 0.5 in TSB, and 10 *μ*l cell suspension (∼10^4^ CFU/ml) was added to 96-well plates. 180 *μ*l TSB containing thymol solution was also added to each well to obtain final concentrations of 0, 9.4, 37.5, 75.0, and 150 *μ*g/mL. All plates were placed in a humidified incubator at 37°C for 24/48 hours. Centrifugal 96-well plate and lower ambient temperature are helpful in eliminating steam influence on test results before test [43].

### 2.5. Determination of Membrane Destruction and Depolarization

PI staining was used to indicate damage to the cytoplasmic membrane, which penetrates only when there is significant damage to membrane. *S. aureus* cultures at mid-exponential phase were collected by centrifugation and suspended in PBS to the final concentration of ∼10^5^ CFU/mL. PI staining solution was added to the cell suspension, and the final concentration is 1 *μ*g/mL. The mixtures were incubated in darkness at 37°C for 10 min and then divided into the wells of a 96-well plate. Thymol in different concentrations with PBS containing 2.5% ethanol was added to the wells and incubated for 30 min at 37°C. The fluorescence values of cell samples were measured every 60 s for 10 min by using a microreader with the excitation wavelength 536 nm and emission wavelength 617 nm. At the same time, cells with cytoplasmic membrane lesion were also evaluated by using a flow cytometer (Beckman Cyto-FLEX FCM) with a blue argon laser at 488 nm. A control group without thymol treatment was also labeled with PI, and a similar test was performed.

Abcam's Cellular Membrane Potential Assay Kit (Fluorometric-Orange) (ab176764) is a homogeneous assay with fast read time and uses a proprietary membrane potential indicator to detect the membrane potential change that is caused by the opening and closing of the ion channels. These cells were obtained in accordance with the method described in Section 2.2, then evenly mixed with the prepared MP Sensor Dye-loading solution in the 96-well plate, and incubated at room temperature for 45 min. Finally, the 96-well plate was placed in a multiwell spectrophotometer to detect the fluorescence intensity at the wavelength of *E*_*x*_/*E*_*m*_ = 530/570 nm.

### 2.6. Determination of Intracellular NADP^+^/NADPH

Intracellular NADPH was detected using an NADP+/NADPH assay kits (MAK038-1 KT, Merck KGaA, Darmstadt, Germany). According to the protocol for collection of *S. aureus* ATCC25923, and five titers of thymol solution addition (0, 0.5MIC, 1.0MIC, 1.5MIC, and 2.0MIC) with PBS containing 2% ethanol, homogeneous samples were obtained by washing, precipitation, preliminary extraction, and other multistep treatment and then treated with either 100 *μ*L of NADP^+^ extraction buffer for NADP^+^ determination or 100 *μ*L of NADPH extraction buffer for NADPH determination. Finally, read fluorescence intensity at *λ*_ex_ = 530 nm/*λ*_em_ = 585 nm for time “zero” and after a 30-minute incubation at room temperature and plate was protected from light during this incubation.

### 2.7. Scanning Electron Microscopy Analysis

Scanning electron microscopy (SEM) analysis was performed to determine the mode of action of thymol on *S. aureus* ATCC25923 as described in Zhou et al. (2019) [44]. After 6.0 h treatment with different concentration of thymol, the *S. aureus* strains were harvested by centrifugation for 10 min at 500 g, washed twice with phosphate buffered saline (1XPBS), and resuspended in PBS containing 2.0% glutaraldehyde to fix the cells. After 1.5 h fixation at 4°C, the cells were washed with Milli *Q* water and then dehydrated in a gradient alcohol concentration (25%, 50%, 75%, 90%, and 100%) for 10 min at each concentration. Finally, the dehydrated samples were sputter coated with gold under vacuum and then observed under a Quanta 200 scanning electron microscope (FEI, USA), at an accelerating voltage of 15 KV and a magnification of 8000×. Control samples without thymol treatment were also prepared and examined as mentioned above.

### 2.8. Determination of Lipid Peroxidation

We harvested the number of cells needed for each assay (∼2 × 10^6^ cells) and washed cells with cold PBS after we mixed 300 *μ*L of MDA Lysis Buffer with 3 *μ*L BHT (100X). Then, homogenized cells were put in 303 *μ*L Lysis Solution (Buffer + BHT) using a Dounce homogenizer (10–50 passes) on ice. When 70–80% of the nuclei do not have the shiny ring, centrifuge at 13,000× g for 10 minutes to remove insoluble material and collect supernatant into 1.5 ml centrifuge tubes. Next, 600 *μ*L of TBA reagent was added into each well containing 200 *μ*L standard and 200 *μ*L sample and incubated at 95°C for 60 minutes. Finally, cool to room temperature in an ice bath for 10 minutes, measuring absorbance immediately on a microplate reader at OD 532 nm for colorimetric assay and RFU at *E*_*x*_/*E*_*m*_ = 532/553 nm for fluorometric assay.

Concentration of MDA in the test samples is calculated as

(1) $$\begin{array}{c} \text{MDA Concentration}=\left(\frac{A}{mL}\right)*B*C=\frac{\text{nmol}}{mL}, \end{array}$$

where *A* = Amount of MDA in sample calculated from the standard curve (nmol); mL = Original plasma volume used (0.020 mL); *B* = Correction for using 200 *μ*L of the 800 *μ*L Reaction Mix; *C* = Sample dilution factor.

### 2.9. Statistical Analysis

All experiments were done in triplicate and repeated at least twice to ensure data credibility. The software R-4.1.0 was used for data analysis. Data were presented as the mean value ± standard deviation (*n* = 3), and differences between groups were tested by Student's *t*-test.

## 3. Results and Discussion

### 3.1. Inhibition Effect of Thymol against *S. aureus*

Thymol, a noncolor and crystalline monoterpene phenol, is a terpenoid with a hydroxyl group on the phenolic ring (Figure 1(a)). Various pharmacological functions, such as antioxidant, anti-inflammatory, and effective against bacterial and fungal species, were reported in previous studies. Many researchers have shown the antibacterial action of this phenolic compound due to its ability to cause structural and functional damage to the cytoplasmic membrane [44]. However, the exact mechanism of its bactericidal activity is not known. To identify the potential roles of thymol, we firstly explored inhibitory effect of thymol against *S. aureus*. As shown in Figure 1(b), thymol at a concentration of 300 *μ*g/mL showed an effective inhibitory effect on *S. aureus* ATCC25923. Consistently, previous studies reported that the min inhibitory concentration of thymol against *S. aureus* ATCC25923 was 0.2 mg/mL [44]. To further explore the inhibitory effect of thymol against the growth of *S. aureus* ATCC25923, we just cultured the *S. aureus* with thymol at the concentrations of 9.4, 37.5, 75.0, and 150.0 *μ*g/mL in the growth curve assays. Atcc43300+ is relatively stable at different concentrations, which is attributed to the fact of being the standard strain of methicillin resistance. Such characteristic makes it perform better than the other three flora. As shown in Figure 1(c), during the 48-hour cultivation process, thymol at the concentration 150 *μ*g/mL inhibited the growth of *S. aureus* within 48 h, while thymol at the concentration 75 *μ*g/mL also revealed a certain inhibitory effect. And we found that, after reducing the concentration of thymol, the time for *S. aureus* to reach the stationary phase was also shortened by 1–4 hours. Those results suggested that thymol can inhibit the growth of *S. aureus* ATCC25923 at low concentrations.

### 3.2. Cell Membrane Damage in *S. aureus*

It was previously reported that thymol is effective against Xanthomonas and has been demonstrated due to increased ROS and activation of apoptosis related proteins [45]. Tian et al. [46] had reported that thymol broke the cell membranes and disrupted intracellular homeostasis in *E. sakazakii* [46]. Therefore, Flow Cytometry and Scanning Electron Microscopy were employed to study whether thymol can also cause damage to the cell membrane of *S. aureus* to achieve its antibacterial activity. The supernatant was stained and analyzed with the PI kit. Obviously, the cell membrane of *S. aureus* was damaged after being treated with thymol for 6 hours (shown in Figure 2(a)). Compared with the control group, the rate of cell membrane damage increased from 0.26% to 7.82% with 500 *μ*g/mL. In order to further verify such phenomenon, we used Scanning Electron Microscopy to analyze the cell membrane damage before and after thymol treatment. As shown in Figure 2(b), after thymol treatment within 6 hours, the cell membrane of *S. aureus* developed an inward trap, and some of the cell membranes were even completely damaged. In Figure 2(a), cells were alive in some extent. Hence, the distribution of such cells was more concentrated than that in Figure 2(b). The number of cells with membrane damage is almost half of the total cells (Figures 2(b) and 2(c)). Membrane potential depolarization is a sign of membrane damage. This means that the polarized cells without drug treatment produce low signals, while the depolarized cells exhibit enhanced fluorescence [46]. Abcam's cell Membrane Potential Assay Kit was used to follow the membrane potential change when thymol is administered. The result in Figure 2(d) showed that when the concentration of thymol reached 500 *μ*g/mL, the membrane potential increased significantly (*p* < 0.005), and the concentration of thymol at 300 *μ*g/mL and 200 *μ*g/mL also revealed a noticeable increase. These results suggested that this mechanism of action of thymol might lead to membrane potential depolarization in *S. aureus*, resulting in membrane damage and bacterial cell death.

### 3.3. Thymol Disrupted Intracellular Homeostasis

The NADP^+^/NADPH and ATP levels in intact cells are in a stable state. However, the destruction of cell homeostasis and integrity may cause changes in intracellular NADP^+^/NADPH and ATP under stress [47–50]. We have previously shown that thymol can cause cell membrane damage in *S. aureus*, but why thymol has such a strong membrane damage ability was not clear. Therefore, it is worthwhile to further study the depolarization and damage effects of thymol. First, we used the NADP^+^/NADPH detection kit to follow the changes in the concentration of NADPH in *S. aureus* cells after thymol treatment for 6 hours. As shown in Figures 3(a) and 3(b), when *S. aureus* was treated with thymol for 6 hours, the concentration of NADPH in the cytoplasm was greatly reduced. But compared with the original level, the concentration of NADP^+^ was increased by 1.5 times. When the value of thymol concentration is 0, the cells are survived as usual. It has the weakest signal strength. And in the condition of 500 *μ*g/ml, the intracellular homeostasis is destroyed seriously. So, it has the largest volume of expansion and production increase. The difference of axis 0 and 500 is the largest. The ATP bioluminescence method was designed to assessed the effect of thymol on intracellular ATP concentrations. The intracellular ATP concentrations in *S. aureus* decreased after 300 *μ*g/mL and 500 *μ*g/mL thymol treatment compared with the control group, while no conspicuous variation was found in 50 *μ*g/mL and 100 *μ*g/mL thymol treated cells. In summary, our result demonstrates that 300 *μ*g/mL and 500 *μ*g/mL thymol cause an increase in NADP^+^ and a decrease in cytoplasmic NADPH and ATP concentration in *S. aureus*, which indicated the possible leakage of intracellular components induced by the thymol and the disruption of the physiologically NADP^+^/NADPH balance.

### 3.4. Loss of NADPH Is Major Cause of Cell Death

NADPH is essential in unremitting flux of energy process due to its ability to serve as electron carriers for a large subset of oxidoreductases [51]. For example, in fed rat livers, the cytosolic free NADP^+^/NADPH ratio is about 0.01, which is mostly in the reduced form to drive reductive biosynthesis reactions [52]. NADPH plays a key role in cellular antioxidation systems by providing reducing equivalents to generate reduced forms of antioxidant molecules to overcome the cytotoxicity and lead to DNA damage and cell apoptosis [53]. *S. aureus* cells were cultured in the TSB culture medium containing thymol with 150 pmol of NADPH or ATP to study the effect of thymol on cell viability. Compared with the control group, normal cells incubated with NADPH and thymol showed a significant increase in cell viability, while cell viability did not change in the ATP and thymol groups. More importantly, we found that NADPH did not completely remove the bacteriostatic effect of thymol but effectively alleviated this role (Figure 4(a)). The heat-treated cells have lost their original cell viability. No matter how thymol is mixed with ATP or NADPH, the biological viability of the cells cannot be restored (Figure 4(b)). We also found that the addition of NADPH only alleviated but did not remove the inhibitory effect of thymol (Figures 4(a) and 4(b)). There are two factors that we think are worth considering: the first is that the effective concentration of NADPH decreases after a period of time due to the continuous consumption of NADPH, and the other is that thymol may exert its antimicrobial effect through other pathways. In a subsequent work, we tracked the changes in the growth curve of *S. aureus* within 24 hours after administration of NADPH and measured the contribution of NADPH in the antibacterial effect of thymol. In keeping with the results of previous studies, when thymol and NADPH are cocultured at the same time, the addition of NADPH can ease cell growth stress and improve cell growth state regardless of the concentration of thymol at 100 or 200 *μ*g/mL. In summary, our results showed that thymol administration process will make the cells lose large amounts of NADPH, which is the cause rather than the result of cell membrane polarization and cell death. Although the concentration of ATP has decreased, ATP cannot effectively alleviate the loss of cell viability caused by thymol. This phenomenon indicates that ATP concentration balance may play an important role in other processes such as maintenance of cell membrane potential and energy supply [46, 54, 55].

### 3.5. NADPH Reduces the Oxidation of Membrane Lipids Caused by Thymol

Lipid peroxidation and leakage of cytotoxic enzymes from lysosomes are important intracellular sources of plasma membrane damage in physiological states, and lipid peroxidation is further exacerbated upon reoxygenation [56]. Thymol disturbs the balance of the important reducing power NADPH concentration in cells, and what confuses us is that there is no direct evidence that NADPH depletion causes lipid peroxidation. To find out whether thymol caused the oxygenation of cell membrane lipids, according to the principle that the higher the degree of lipid oxidation is, the higher the concentration of malondialdehyde (MDA) is generated, the change of MDA concentration is used as an indicator to track the oxidation level of cell membranes. Consistent with our conjecture, when the concentration of thymol reached 300 *μ*g/mL or 500 *μ*g/mL, the soluble MDA concentration reached 0.4 nmol/mL and 0.5 nmol/mL respectively, and there was a significantly increased difference compared with 0.1 nmol/mL in the control group. It is worth noting that, within the 100 *μ*g/mL concentration range, the observed upward trend is not very prominent (Figure 5(a)). For further administration of 150 pmol of NADPH into TSB containing thymol to reduce the cell membrane oxidation level, we were pleasantly surprised to find that 150 pmol NADPH was fully sufficient to recover the cell membrane peroxidation caused by 200 and 300 concentrations of thymol. However, this recovery failed to adjust the normal physiological level, which may be due to the decreased physiological activity of the cell after the damage of the cell membrane. Another possible reason is that the repair pathway equipped with the cell did not restore the integrity of the membrane.

In this part, we subsequently employed the Scanning Electron Microscopy to detect the effect of NADPH on cell membrane trap generation and development. The *S. aureus* strains were firstly treated with 300 *μ*g/mL of thymol at 37°C and then were collected by centrifugation for 10 min at 4000 g. The collected cells were fixed and dehydrated in the process described in Section 2.7. Finally, the samples were analyzed under scanning electron microscope. As shown in Figure 5(c), the number of cell membrane traps formed on membrane of *S. aureus* after the addition of NADPH and thymol was fewer, and the diameter of the traps also showed a visible decrease compared with that treated with thymol alone (Figures 2(c)-2(d) and 5(c)-5(d). To sum up, our in vitro experiment and SEM results suggested that NADPH was depleted as a result of the cell membrane lipid oxidation levels increase. However, a certain amount of NADPH supplementation does not completely alleviate the peroxidation reaction, nor does it completely reduce the number and size of cell membrane traps.

### 3.6. NOX_2_ Is Involved in Cell Membrane Damage Induced by Thymol

Although it has been previously stated that thymol induces cell membrane damage because of NADPH depletion, how NADPH in cells transfers to NADP^+^ is still unknown. In order to more clearly explore the antibacterial effect of thymol, we further analyzed whether several NADPH-related kinases were involved in thymol-induced cell membrane damage. Our unpublished results and other published papers suggest that NOX_2_-catalyzed oxidation of NADPH to form peroxide free radicals is a possible factor in NADPH depletion. We then used Western blot to detect the expression level of NOX_2_ when the *S. aureus* was treated within thymol. After thymol treatment for 6 hours, the expression level of NOX_2_ shows a positive correlation with the concentration of thymol [57, 58]. As shown in Figure 6(a), NOX_2_ expression increased nearly fourfold after treatment with 300 *μ*g/mL thymol compared with 100 *μ*g/mL sample. Next, we used si-RNA silencing to knock down the expression of NOX_2_ in *S. aureus* to observe the effect of NOX_2_ on cytoplasmic NADPH and NADP ^+^ concentration. We were pleasantly surprised to find that when NOX_2_ was knocked down, and *S. aureus* was treated with thymol, the concentration of soluble NAPH in the cytoplasm was significantly increased compared to the control (Figure 6(c)). And we also found that there was a significant decrease in the concentration of NADP^+^. These results directly indicate that thymol can change or destroy the morphology of the cell membrane by changing the concentration of NADPH/NADP^+^ in the cytoplasm, thereby mediating the death of *S. aureus*. And Figure 7 is the Graphic abstract of this paper.

## 4. Conclusion

The growth of *S. aureus* can be effectively inhibited by thymol, which is firstly confirmed in this paper. Furthermore, the inhibitory concentration of thymol is also measured by Broth Micro-Dilution method. Thymol might lead to membrane potential depolarization in *S. aureus*, resulting in membrane damage and cell death. In order to further understand the corresponding antibacterial mechanism, the concentration of soluble NADP^+^/NADPH and ATP in the cytoplasm is detected. Thereafter, an increase in NADP^+^ and a decrease in cytoplasmic NADPH and ATP are caused by thymol. Such phenomenon indicated the possible leakage of intracellular components and the disruption of the physiologically NADP^+^/NADPH balance. Then, the biochemical experiments and SEM results suggested that the cell membrane lipid oxidation levels are significantly increased by using thymol treatment. Besides, a certain amount of NADPH supplementation can not completely alleviate the peroxidation reaction and reduce the number and size of cell membrane traps. The restricted catalytic enzyme NOX_2_ can regulate the balance of NADPH/NADP^+^. So, NOX_2_ can be a potential downstream target of thymol in the cell. Finally, a specific guidance is provided in food preservation and storage about the use of thymol.

## Figures and Tables

**Figure 1:** Thymol inhibits the growth of *S. aureus* . (a) Chemical structure of thymol. The main structure is a benzene ring, containing three methyl groups (CH_3_) and one hydroxyl group (OH). (b) Inhibitory effect of thymol against *S. aureus*. The standard concentration of thymol (1200 *μ*g/mL) was prepared firstly, and then we used progressive dilution method to get culture medium with the final concentrations of 50, 100, 150, 200, 300, 400, 600, and 800 *μ*g/mL, respectively. (c) The growth inhibition of thymol against *S. aureus*. The strain was cultured for 6 hours in the medium containing 0, 9.4, 37.5, 75.0, and 150 *μ*g/mL thymol, and the OD600 values were determined by microplate reader.

**Figure 2:** Thymol treatment resulted in cell membrane destruction. (a)-(b) *S. aureus* were first collected into a 15 mL centrifuge tube and then washed twice with precooled 1 × PBS solution. After centrifugation at 500× g for 3 minutes, the supernatant was discarded to collect the cells, and 300 *μ*L binding buffer was added to adjust the cell concentration to 10^6. Gently mix it with 5.0 *μ*L Annexin-V and 10 *μ*L PI, incubate it at 37°C for 15 min, and protect it from light. The selected detection channel is 488 nm, the acquisition band is 530 nm/30 nm, PI: 561 nm, and the acquisition band is 610 nm/20 nm. (c) Scanning electron microscope pictures of *S. aureus* without thymol treatment (left) and thymol treatment (right). (d) The number of cells with normal cell membrane morphology and the number of cells with damaged cell membrane morphology in the field of the scanning electron microscope; each experiment was repeated three times.

**Figure 3:** Thymol disrupted intracellular homeostasis. (a) Changes in cell membrane potentials of *S. aureus* treated with different concentrations of thymol. (b)-(c) The concentration of soluble NADPH (b) and NADP^+^ (c) in the cytoplasm was tested by the kit, and samples of *S. aureus* treated with thymol for 6 hours and control samples were obtained by centrifugation. These samples were then measured according to the method described in Section 2.6. (^*∗∗∗*^*p* < 0.001). (d) The intracellular ATP concentrations in *S. aureus* decreased after 300 *μ*g/mL and 500 *μ*g/mL thymol treatment. All experiments were repeated three times.

**Figure 4:** The increase in cell viability is due to NADPH administration. The cells were incubated with thymol and NADPH/ATP for 6 hours, and the changes of cell viability were determined by using a dedicated cell activity detection kit. All tests were performed according to the instructions in the kit. Results of cellular viability of wild-type normal cells without any treatment (a) and heat-treated cells (b). (c) Growth curves for *S. aureus* cultured in TSB containing 100/200 *μ*g/mL thymol and 150 pmol NADPH. NADPH partially dissolves the inhibitory effect of thymol on bacterial growth.

**Figure 5:** NADPH reduces the oxidation of membrane lipids. The higher the degree of lipid oxidation is, the higher the concentration of malondialdehyde (MDA) is generated in cells. (a) Cell membrane oxidation levels of thymol treated cells were measured in vitro. (b) When treated with NADPH and thymol simultaneously, the lipid oxidation level of cell membrane was determined. (c) Scanning electron microscope images of cells treated with 0 *μ*g/mL thymol + 150 pmol NADPH (left panel) or 300 *μ*g/mL thymol + 150 pmol NADPH (right panel). (d) The number of normal and damaged cells calculated from the microscope photograph.

**Figure 6:** NOX_2_ is involved in NADPH/NADP ^+^ balance adjustment. (a) We used Western blot to detect the expression of NOX_2_ protein in *S. aureus* ATCC25923. (b) RNA interference and Western blot methods were used to study the effect of knockdown of NOX_2_ expression on the effect of thymol in *Staphylococcus aureus* (+100 *μ*g/mL). (c) After knocking down NOX_2_, when *S. aureus* is treated with thymol, the concentration changes of NADPH/NADP^+^ in the cytoplasm.

**Figure 7:** Graphic abstract.

## Data Availability

The experimental data used to support the findings of this study are available from the corresponding author upon request.
